# Diagnosis of Breast Cancer Using Computational Intelligence Models and IoT Applications

This article has been retracted.

**DOI:** 10.1155/2022/2143510

**Published:** 2022-10-14

**Authors:** Mohammed Alghamdi, Mohammed Maray, Malik Bader Alazzam

**Affiliations:** ^1^College of Computer Science, King Khalid University, Abha 62529, Saudi Arabia; ^2^University of Jeddah, Jeddah, Saudi Arabia; ^3^Information Technology College, Ajloun National University, Ajloun, Jordan; ^4^The University of Mashreq, Research Center, Baghdad, Iraq

## Abstract

The use of computer-aided diagnostic (CAD) models has been proposed to aid in the detection and classification of breast cancer. In this work, we evaluated the performance of multilayer perceptron neural network and nonlinear support vector machine models to classify breast cancer nodules. From the contour of 569 samples, ten morphological features were used as input to the classifiers. The average results obtained in the set of 50 simulations performed show that the proposed models showed good performance (all exceeded 90.0%) in terms of accuracy in the test set. The nonlinear support vector machine algorithm stands out when compared to the proposed multilayer perceptron neural network algorithm, with 99% accuracy and a 2% false-negative rate. The neural network model presented lower performance than the nonlinear support vector machine classifier. With the application of the proposed models, the average results obtained are promising in the classification of breast cancer.

## 1. Introduction

Cancer has become one of the most frequent diseases in the world, accounting for 15 percent of the almost 56 million deaths, with more than 14 million new cases annually [1]. In Iraq, estimates for 2018 point to more than 600,000 new cancer cases, where breast cancer is the one with the highest incidence, after nonmelanoma skin and prostate cancer [2, 3]. Since the beginning of research on breast cancer, the best way to cure of the disease is early detection. Mammography is one of the best techniques for screening breast cancer currently available, capable of recording images of the breast in order to diagnose the presence or absence of structures that may indicate the disease. With this type of exam, the tumor can be detected before it becomes palpable. However, the evaluation of the mammography exam and the diagnosis, performed by a radiologist, requires a lot of skill, but there are limitations in the primary prediction of breast cancer. Studies have revealed that 10% to 30% of women who have had breast cancer have negative results when undergoing mammography, which leads to the belief that there was a misinterpretation of the exams. Distortions in the interpretation and classification of lesions by specialists imply a greater number of unnecessary biopsies, that is, between 65% and 85% of breast biopsies are performed in benign lesions. As a result, there is a reduction in the cost-effectiveness of the tests and, in the worst case, the nondetection of the disease, characterizing a false-negative diagnosis. This neoplasm has attracted greater attention in public health and the scientific community, where researchers are using computational intelligence techniques to develop computer diagnostic support systems (CAD), aiming to increase the detection rate of breast cancer [4]. Among these techniques, Artificial Neural Networks (ANNs) [5, 6] and Support Vector Machines (SVMs) [7], because they are robust in a noisy dataset. Despite the good results obtained with ANNs, their results are stochastic and strongly depend on the order of presentation of objects and the initial weights assigned to their connections. Therefore, it is recommended to run it several times for different configurations of the data and initial values of weights, obtaining an average of performance the Nonlinear Layers (NLPs) and Support Vector Machine (SVM) in a set of 50 simulations in the classification of breast malignancy, obtained from mammographic findings.

## 2. Theoretical Framework

Artificial Neural Networks (ANNs) are parallel and distributed systems made up of simple units (neurons or nodes), which calculate certain mathematical functions (mainly nonlinear) and have the capacity for generalization, self-organization, and temporal processing. Similarly to the nervous system of a human being, neurons are arranged in one or more layers and interconnected by numerous connections, usually unidirectional, called synapses [8, 9]. These connections are associated with values, called synaptic weights, responsible for weighing the inputs of each neuron as a way of storing knowledge of a particular model. Artificial neurons, also known as nodes, or processing units, are used in neural networks to facilitate learning.  Figure 1 shows a representation of the nonlinear model of an artificial neuron.

An ANN has the characteristic of learning through examples and extracting knowledge from a given data set. Knowledge is acquired from the process by which the free hyperparameters of a neural network are adjusted through a continuous form of stimulation by the external environment, aiming to minimize the value of an error function. This process is defined as learning, which can be classified as supervised or unsupervised. Within the supervised learning context, we present the available inputs and the desired output to the network, and the algorithm works to adjust the synapse weights by calculating the difference between the desired output value *y*_di_(*t*) and the value predicted by the ANN *y*_pi_(*t*), at instant *t* thus producing an error *δ*(*t*) in the following equation:

(1) $$\begin{array}{c} \delta \left(t\right)=y_{di}\left(t\right)-y_{pi}\left(t\right)\text{.} \end{array}$$

The generic way to adjust the weights, by error correction, is presented in the following equation:

(2) $$\begin{array}{c} w_{ij}\left(t+1\right)=w_{ij}\left(t\right)+\eta \;e_{i}\left(t\right)x_{i}\left(t\right)\text{,} \end{array}$$

where *η* is the learning rate and *x*_*i*_(*t*) the input to neuron *i* at time *t*.

In unsupervised learning, the desired output values *y* di are not known. Therefore, learning occurs through the identification of patterns in the inputs. The choice of an ANN architecture is related to the types of problems to be addressed and is defined by 4 main hyperparameters: number of network layers, number of neurons in each layer, type of connection between neurons, and the network topology. Regarding the number of layers, there are single-layer networks, which have only one node between the input and output layers of the network, being restricted to solving linearly separable problems.

Multilayer neural networks have more than one neuron between an input and an output of the network. Among the multilayer networks, we have the Multilayer Perceptions (MLP) type, which has one or more layers of intermediate or hidden neurons and is considered a universal approximator. According to the universal approximation theorem, any continuous function can be uniformly approximated by a network with at least one layer of hidden neurons and a sigmoid activation function [9]. Let *φ*(.) be a continuous, bounded, and monotonously function *I*_mo_ and a unitary hypercube 0,1]^mo^ of dimension mo. The space of continuous functions on *I*_*mo*_ is represented by C *I*_mo_. Then, given any function *f*∋ C (*I*_mo_) and *ε*  >  0, there is an integer *M* and sets of real constants *α*_*i*_, *b*_*i*_ and *w*_*ij*_, where *i*=1, . . . ,mi and *j*=1, . . . , mo such that we can define:

(3) $$\begin{array}{c} F\left(x_{i}\ldots ,x_{mo}\right)=\overset{m1}{\underset{i=1}{\sum }}\alpha_{i}\varphi \left(\overset{m0}{\underset{j=1}{\sum }}w_{ij}x_{j}+b_{i}\right)\text{.} \end{array}$$

An approximation to the function *f*(.) is shown in 2.3,

(4) $$\begin{array}{c} \left|\left.{F\;\left(x\right.}_{1}\ldots ,\left.x_{mo}\right)-{F\;\left(x\right.}_{1}\ldots ,x_{mo}\right)\right|-\varepsilon \text{.} \end{array}$$

For (*x*_1_ …, *x*_mo_) everything in the input space.

So the universal approximation theorem is directly applicable to multilayer perceptrons.  Figure 2 represents an MLP network with three inputs, two intermediate layers with four neurons, and an output layer with one neuron, producing single output information [10].

MLP networks have been successfully applied to solve several problems, through their training in a supervised way using the error backpropagation algorithm, which has two distinct phases. In the first phase, the functional signal propagates (feedforward) keeping the weights fixed to generate an output value from the inputs supplied to the network. In the second phase, the outputs are compared with the desired values, generating an error signal that propagates from the output to the input, adjusting the weights to minimize the error [11, 12]. Thus, the way to calculate the error depends on the layer in which the neuron is located, as shown in the following equation:

(5) $$\begin{array}{c} \delta_{l}=\left\{f_{a}^{\prime }\right)e_{l}\;f_{a}^{\prime }\sum w_{lk}\delta_{k}\;if\;n_{l}\in C_{sai}\;n_{l}\in C_{int}\text{,} \end{array}$$

where *n*_*l*_ is the *l*^th^ neuron, *C*_sai_ represents the output layer, *C*_int_ represents an intermediate layer, is the partial derivative of the neuron's activation function, and el is the squared error made by the output neuron when its response is compared to the desired, which is defined by the following equation:

(6) $$\begin{array}{c} e=\frac{1}{2}\overset{k}{\underset{q=1}{\sum }}{\left(y_{q}-{\hat{y}}_{q}\right)}^{2}\text{,} \end{array}$$

where ${\hat{y}}_{q}$ is the output produced by the neuron and *y*_*q*_ is the desired output.

The partial derivative defines the adjustment of the weights, using the gradient descent of the activation function. This derivative evaluates the contribution of each weight in the network error to the classification of a given object. If the derivative for a given weight is positive, the weight is causing the difference between the network output and the desired output to increase. Therefore, its magnitude must be reduced in order to decrease the error. Otherwise, the weight will contribute to the network output being closer to the desired one.

The Support Vector Machine (SVM) is a set of supervised learning methods used for data classification and regression based on statistical learning theory. Algorithms have qualities that allow them to generalise to previously unexplored data sets. Creating a border between two classes permits the prediction of labels from one or more feature vectors [13]. Using a hyperplane as a decision boundary, all data points near each class are placed as close to the boundary as possible. Support vectors are the names given to the closest points in space. Consider a training dataset that is labelled like this:

(7) $$\begin{array}{c} \left(x_{1}\;,y_{1}\right),\ldots \left(x_{n}\;,y_{n}\right),x_{i}\in R^{d}and\;y_{i}\in \left(-1,+1\right)\text{,} \end{array}$$

where *x*_*i*_ is a representation of the feature vector and *y*_*i*_, Negative or Positive Class Label of a Training Set It is thus possible to define the ideal hyperplane:

(8) $$\begin{array}{c} wx^{t}+b=0\text{,} \end{array}$$

where *w*, *x*, and *b* represent the input and trend, respectively (or bias). All elements of the training set must meet the following inequalities:

(9) $$\begin{array}{c} \begin{array}{c} wx_{i}^{t}+b\geq 1,\;if\;y_{i}=1,\\ wx_{i}^{t}+b\leq -1,\;if\;y_{i}=-1. \end{array} \end{array}$$

In order to train an SVM model, the goal is to discover the *w* and *b* that maximise the margin 1/||*w*||^2^in the hyperplane.

Thus, for a linearly separable dataset, SVMs are able to categorize two classes through an optimal hyperplane, obtaining a good generalization in its classification. However, for binary classification, where the data are not linearly separable in the original space, it is necessary to reference it in a new space of greater dimension, called feature space. For this, the use of nonlinear Support Vector Machines (nonlinear-SVMs) is necessary.

This type of approach is called nonlinear support vector machines (SVMs-nonlinear), and it is used to classify data represented in multidimensional feature space by the kernel function. SVMs use the kernel function to transform nonlinearly separable data into linearly separable data in a higher-dimensional space. These functions convert the dataset into the feature space's original input space, i.e., a *K* kernel takes two input space points *x*_i_ and *x*_j_ and returns the feature space's dot product. Kernels are incorporated into the SVMs classifier through the following equation:

(10) $$\begin{array}{c} f\left(x\right)=sgn\left(\overset{n_{SV}}{\underset{i=1}{\sum }}\alpha_{i}y_{i}K\left({\overset{⟶}{x}}_{i},\overset{⟶}{x}\right)+b\right)\text{,} \end{array}$$

where *K* denotes the kernel function, which receives as input the support vector *i* and the sample values to be classified, *α i* the Lagrange multipliers and *b* the intercept value.

Methods based on kernel theory have provoked a real revolution in the algorithms of statistical learning theory, supervised and unsupervised, by enabling the creation of nonlinear versions of classical linear algorithms. Among the set of algorithms found in the literature that use kernel function, the support vector machine algorithm proposed by Vapnik 20 for binary classification is the most prominent. SVMs have kernel functions that characterize their pattern recognition mode, with polynomial, Gaussian, and sigmoidal being the most used (Table 1).

The degree (*δ*) can be defined during training in the polynomial function. In the Gaussian function that corresponds to an infinite-dimensional feature space, its use allows SVMs to present a radial basis function (RBF) neural network characteristics. The sigmoidal function allows behavior similar to that of an MLP neural network. SVMs use a decision function to distinguish between two groups of data (hyperplane). We refer to the points taken from the training data as support vectors (SVs). Unlike classic pattern recognition methods, SVMs focus on reducing structural risk rather than empirical risk.

## 3. Materials and Methods

The Wisconsin Diagnostic Breast Cancer public database 21 provided the data for this investigation, which included 569 records from women with probable breast cancer. Mean values of radius, texture, perimeter, and area are included in the data analysis, the number of concave points in the contour, and the fractal dimension of the lesion's contour. The methodology aims to compare the computational models structured in Neural Network MLP and Support Vector Machines (SVMs-nonlinear), in the classification of malignancy, referring to the morphological characteristics of the contour of the lesion found in mammographic findings (Figure 3).

To evaluate the performance of the models proposed in this study, the total accuracy or precision (ACC) and the error rate of the false-negative class (EFN) were used. Defined, respectively, by the following equation:

(11) $$\begin{array}{c} \begin{array}{c} Accuracy\left(ACC\right)=\frac{VP+VN}{n}\\ False-negative\;class\left(EFN\right)=\frac{FN+VN}{VP+FN} \end{array} \end{array}$$

where V P are positive-label samples (+1) predicted to be positive, V N are negative-label samples (−1) predicted to be negative, F N are positive-label samples (+1) predicted to be negative, and *n* is the total number of samples. For each model, 50 simulations were performed to obtain a better generalization in the results obtained.

The computational models were implemented using the R software and the Kernlab13 and Neuralnet6 packages, respectively, in the SVMs-nonlinear model and in the MLP neural network model. The list of hyperparameters used in the RN-MLP and SVMs-nonlinear models is summarized in Tables 2 and 3, respectively. The hyperparameters used in the classification were obtained empirically.

## 4. Results and Discussions

The computational models proposed in this work were evaluated by incorporating attributes referring to the radius, texture, perimeter, area, smoothness, compactness, concavity, several concave points in the contour, symmetry, and fractal dimension of the lesion from the data set of patients with mammary microcalcification. The average results obtained in the 50 simulations with the application of the models are represented in Tables 4 and 5.

The RN-MLP model, in its best simulation, obtained an accuracy of over 94%, with a false negative value of 2%. Indicating an accuracy of 98% in terms of sensitivity in the test set. Regarding the error in false-negative detection, the model obtained an average value of less than 10% in the set of 50 simulations performed.

According to the analysis of the results presented in Table 5, it is possible to verify the promising performance of the SVM-nonlinear structured model. In its best simulation, an accuracy above 98% and a false negative error rate of less than 2% (1.96%) were obtained. Regarding the leave-one-out (CVE) cross-validation error, we can verify that it obtained an amplitude between the maximum and minimum value obtained of 4% in the 50 simulations performed. The average results obtained by the RN-MLP and SVM-nonlinear models, in the categorization of malignancy in the set of simulations performed, is represented in Table 6.

To select the best and worst simulation, the value of the false-negative error obtained by the models was used, since this hyperparameter is of paramount importance in categorising malignancy. Applying the test of comparison of means with *p-value*≈0.05, it is possible to verify the existence of a statistically significant difference between the results, referring to the accuracy between the models used in the study. Indicating that for the ACC hyperparameter the SVM-nonlinear model has better performance when compared to the RN-MLP model.

Although the SVM-nonlinear model presents a mean value of the false-negative error lower than that obtained by the RN-MLP model, there was no statistically significant difference at the level of 95% (*p*-value≈0.05) among the results obtained by the models. In the 50 (fifty) simulations carried out in the test set, the SVM-nonlinear model obtained a simulation with a value of 100% of sensitivity, that is, 0% in the determination of the false negative error rate. This fact was not verified in the RN-MLP model, where a maximum value of 98% was obtained.

It is important to emphasize that the accuracy obtained by the models, in the classification of breast microcalcification, is close to the values obtained in the literature using techniques based on computational intelligence. Comparing the results obtained by [7], who used the L2-SVM model, in the WDBC classification (ACC≈96.09% and EFN≈2.47%), it can be verified that the model SVM-nonlinear proposed in this study, presented values in terms of accuracy (ACC≈98.59%) and the value of the false negative error rate (EFN≈1.97%) higher.

## 5. Conclusion

The high rate of incidence and deaths caused by breast cancer, currently in Iraq and the world, justify the development of scientific research aimed at strategies to aid in the early detection of the disease, a determining factor for the success of the treatment. In this work, we proposed using computational models structured in RN-MLP and nonlinear SVM to categorize malignancy in mammographic findings. The incorporation of information regarding the morphological characteristics of the contour of the breast lesion, contributed to the performance of the proposed models regarding the determination of the false-negative rate. Therefore, this metric is of paramount importance for health professionals, especially in detecting breast lump malignancy. Despite the results obtained, with the application of the neural network models of multilayer perceptrons and nonlinear support vector machine, the classification of mammary microcalcifications has presented promising results. It is perceived the need to deepen the study. To this end, we intend to develop a hybrid model structured in the future using genetic algorithms and a convolutional neural network to evaluate the performance in the classification of breast lesions and the optimization of the model's hyperparameters.

## Figures and Tables

**Figure 1:** Nonlinear neuron model [9].

**Figure 2:** Graphical representation and an MLP network, with two intermediate layers.

**Figure 3:** Flowchart of the proposed model.

**Table 1:** Mathematical equations regarding the most used kernel functions.

	Function (*k*(*xi*, *xj*)	Parameters
Kernel type	(*δ*(*xi*, *xj*)^*d*^	*δ*, *d* *k*
Polynomial	*e* ^(−*σ*‖*xi*, *xj*‖^2^^	*σ*
Sigmoidal	tanh (*δ*(*xi*, *xj*)+*k*)	*δ*, *k*

**Table 2:** Parameters used in the RN-MLP model.

Parameters	Value
Number of simulations	50
Maximum number of seasons	100000
Activation function	Logistics
Training algorithm	Backpropagation
Metric used in training error	SSE
No. of hidden layers	2
Number of neurons in the first hidden layer	7
Number of neurons in the second hidden layer	4
Initialization of weights	Randomly with values [0, 1]
Stop criterion	0.001

**Table 3:** Parameters used in the SVM-nonlinear model.

Parameters	Value
Classifier type	C-SVM
Kernel function	RBF
Kernel function variance (s)	0.5
*C* Regularization parameter	1
Stop criterion	0.001

**Table 4:** Average performance of the RN-MLP model in categorising malignancy in the set of 50 simulations.

	SSE training error	ACC (%)	EFN (%)
Average ± SD	0.558 ± 0.50	92.58 ± 2.03	9.38 ± 4.39
Average ± irq	0.507 ± 0.94	92.25 ± 3.52	9.49 ± 6.64
Maximum-minimum	1.849-0.022	94.37-89.44	22.22-2.00
Best simulation	0.022	94.37	2

**Table 5:** Average performance of the SVM-nonlinear model in the categorization of malignancy in the set of 50 simulations.

	Error			
	Training error	CVE (%)	ACC (%)	EFN (%)
Average ± SD	3.42 ± 0.53	5.36 ± 0.70	95.8 ± 2.03	9.01 ± 4.46
Average ± irq	3.42 ± 0.70	5.43 ± 0.94	95.8 ± 2.64	8.34 ± 5.2
Maximum-minimum	4.46-2.22	7.249-3.259	98.59-90.84	21.16-0.01
Best simulation	3.52	5.61	98.59	1.97

**Table 6:** Average performance of the models proposed in the study, in the set of 50 simulations.

	SVM-non-linear		RN-MLP	
	ACC (%)	EFN (%)	ACC (%)	EFN (%)
Average ± SD	95.01 ± 1.66	9.01 ± 4.62	92.59 ± 2.07	9.39 ± 4.39
Bad simulation	91.56	21.09	90.86	22.23
Best simulation	98.59	1.97	94.36	2.01

## Data Availability

The data used to support the findings of this study are included within the article.
